# FAMILIAL REACTIVE PERFORATING COLLAGENOSIS

**DOI:** 10.4103/0019-5154.57608

**Published:** 2009

**Authors:** Yasmeen J Bhat, Sheikh Manzoor, Seema Qayoom, Roohi Wani, Asif Nazir Baba, Arshad Hussian Bhat

**Affiliations:** *From the Departments of Dermatology, STD & Leprosy and Pathology, SKIMS Medical, College Hospital, India.*; 1 *From the Departments of Dermatology, SKIMS Soura, Srinagar, India.*

**Keywords:** *Familial*, *umbilicated*, *transepidermal elimination*, *retinoids*

## Abstract

**Background:**

Reactive perforating collagenosis (RPC) is one of the rare forms of transepidermal elimination in which genetically altered collagen is extruded from the epidermis. This disease usually starts in early childhood as asymptomatic umbilicated papules on extremities, and the lesions become more conspicuous with age.

**Aims:**

The objective of our study was to determine the clinico-pathological features of RPC and the response to various treatment modalities.

**Methods:**

Ten patients of RPC, belonging to five different families, were studied clinically. Various laboratory investigations were carried out and diagnosis was made by histopathology of the lesions. Patients were given various topical and oral treatments.

**Results:**

RPC is familial in most cases without any definite inheritance pattern. It begins in childhood and the lesions are usually recurrent and become profuse and large with age. Systemic diseases have no role in the onset of lesions.

**Conclusion:**

Oral and topical retinoids in combination with emollients is the best treatment option.

## Introduction

The perforating dermatoses comprises four varieties: Kyrle's disease, perforating folliculitis, reactive perforating collagenosis, and elastosis perforans serpiginosa. Reactive perforating collagenosis (RPC) is a rare skin disorder characterized by transepidermal elimination (TEE)[1] of altered collagen through the epidermis. TEE is a mechanism by which the skin rids itself of abnormal substance.[2] Two distinct forms of RPC are: the rare inherited form that manifests in childhood, usually precipitated by environmental cold or trauma; and the commonly acquired form that occurs in adulthood and is typically associated with diabetes mellitus and chronic renal failure.[3] Fewer than 50 case reports of the inherited form of RPC exist in the world literature.[4] The basic defect seems to be a genetic abnormality of the collagen leading to its focal damage, which is then extruded as a result of necrolysis of the overlying epidermis. Also, elevated serum and tissue concentration of fibronectin may be responsible for inciting increased epithelial migration and proliferation culminating in perforation.[5]

## Materials and Methods

Ten patients of RPC attending the Dermatology OPD of SKIMS medical college hospital from May 2006 to May 2008 were taken for the study after a written informed consent from them. Clearance was taken from SKIMS review board. The patients were evaluated clinically and the diagnosis was confirmed by histopathology.

A proper history was taken from all the patients with respect to the age, sex, demography, consanguinity among parents, age at presentation, duration, and progression and evolution of lesions. The patients belonged to five unrelated families. Two sisters were involved in first family, brother and sister each in second and third family, father and two sons in fourth family, and only one male in fifth family. Seven patients were born by full-term normal deliveries, whereas three were born by cesarean section, one being preterm. None of the patients had any congenital anomaly. Consanguinity among parents was seen in two patients only belonging to single family. Associated symptoms such as itching, seasonal exacerbation, trauma, mode of birth, and presence of congenital anomalies was specifically investigated. Family pedigree of all the patients was studied. History of involvement of other systems was taken. The clinical examination included the general physical, systemic, and cutaneous examination. The lesions were studied with respect to site, size, number, shape, distribution, morphology, umbilication, atrophy, and scars. Skin biopsy of all the patients was taken for histopathological examination at department of Pathology, SKIMS. Special staining for collagen was done by Verhoeff–van Geison stain. Routine laboratory investigations including blood sugar and renal function tests were carried out.

The patients were tried with various treatment modalities including emollients, topical steroids and retinoids, oral isotretinoin, and vitamin A supplements. Four patients aged more than 12 years at presentation(19, 12, 14 and 38 years, respectively) were put on oral isotretinoin 0.50-0.75 mg/kg/day for a period of 6-12 months. Six patients aged less than 12 years were put on topical tretinoin 0.025% or 0.05% gel with emollients. Oral vitamin A supplements were given to three patients and topical steroid-antibiotics to two patients.

## Results

The group of ten patients comprises five males and five females. The age of presentation ranged from 7 to 38 with a mean of 13.7 years. The age of onset of lesions varied from 1 to 8 years with a mean of 5.3 years. The lesions were itchy only in three patients. Koebner phenomenon in the form of linear lesions was positive in seven patients, whereas cold exacerbation was seen in six patients [Table 1]. In the majority of patients, the lesions began as small, 1-3 mm, asymptomatic, slowly growing, multiple, discrete, asymmetrical, bilateral, skin colored papules on the dorsum of hands. Six patients showed disappearance of the lesions, followed by recurrence in winter season while four had the lesions throughout the year, which progressively increased in size, number and distribution involving face, extremities, and trunk. The lesions developed central umbilication filled with a keratinous plug, became hyperkeratotic and hyperpigmented and caused epidermal atrophy after the plug fell off [Figures 1 and 2]. One patient aged 38 years at presentation showed large giant, intensely pruritic lesions of 10-15 mm size on the face and extremities which healed with scarring, indicating that the lesions become more profuse and enlarged with age unless treatment is given.

**Table 1:** Clinical profile of patients with RPC

Family	Patient no	Age at presentation	Sex	Consanguinity	Age at onset	Koebner phenomenon	Cold exacerbation	Itching	Treatment
One	1	19	F	−	8	+	+	+	Isotre + Em
	2	12	F		8	+	+	−	Isotre + Em
Two	3	9	M	−	1	−	−	−	Tre + St-Ab
	4	14	F		3	+	−	+	Isotre
Three	5	11	M	+	6	+	+	−	Tre + Em + Vit A
	6	8	F		7	+	−	−	Tre + Vit A
Four	7	38	M	−	8	+	+	+	Isotre + Em
	8	9	M		1	+	+	−	Tre + Vit A
	9	7	F		2	−	+	−	Tre + Em
Five	10	10	M	−	7	−	−	−	Tre + St−Ab

Isotre - Oral isotretinoin;  Tre -  Topical tretinoin; Em - Emollient cream; St−Ab - Steroid antibiotic cream;  Vit A - Oral vitamin A supplement

**Figure 1:** Umbilicated erythematous papules on the feet of 12-year-old female

**Figure 2:** Umbilicated hyperkeratotic giant papules with hyperpigmentation and atrophy on the legs of 38-year-old male

None of our patients had any history of diabetes, hepatic, renal, or other systemic involvement, which was confirmed by laboratory investigations. The histopathological examination of all the patients was consistent with reactive perforating collagenosis, showing a central area of depression, parakeratosis, basophilic collagen, and numerous pyknotic nuclei of inflammatory cells [Figure 3]. The epidermis at the base of the plug showed atrophy with perforation through which basophilic bundles of collagen with altered morphology extruded from the dermis, confirmed by Verhoeff- van Geison stain in all patients [Figure 4]. The elastic fibres were normal and seen only in dermis after special staining for elastin, which differentiates it from other perforating disorders.

**Figure 3:** Disruption of epidermis and a central crater containing inflammatory cells and keratinous debris (H and E stain, ×50)

**Figure 4:** Extrusion of collagen fibres (Verhoeff–van Geison stain, ×50)

Treatment response was excellent with oral Isotretinoin in two patients with complete regression of lesions after one year of treatment, while two showed recurrence after three months of cessation of treatment. Topical tretinoin was effective only in smaller lesions and lesions with short duration. Three patients on oral and five on topical retinoids developed xerosis during treatment which was alleviated by emollients. Oral vitamin A supplements did not show any additional improvement, whereas topical steroid-antibiotic creams showed temporary improvement.

## Discussion

Perforating dermatoses comprises four varieties: Kyrle's disease, perforating folliculitis, reactive perforating collagenosis, elastosis perforans serpiginosa.[6] Reactive perforating collagenosis is a rare skin disorder characterized by transepidermal elimination of altered collagen through the epidermis.[7] The two distinct forms of RPC are an inherited form that manifests in childhood and an acquired form that occurs in adulthood. A genetic abnormality of the collagen in upper dermis is suggested as the probable cause for the inherited form of this disorder.[8] The mode of inheritance is not clear. Reports of affected families reveal AD, AR, and sporadic cases.[9] Our study also does not show a single pattern of inheritance. Only two patients from a single family were the products of consanguineous marriage indicating AR inheritance, while in the other family, father and two children were affected indicating AD inheritance.

The lesions of this TEE disorder usually begin in early childhood and the patient may get giant lesions with the increase of age.[10,11] Our patients also developed lesions in early childhood at the mean age of 5.3 years and the lesions became more conspicuous with the increase of age. Pruritus was found only in three patients whose lesions were bigger. Their lesions center residual scarring. Koebner phenomenon was seen in seven patients and the lesions showed exacerbation during winter as reported earlier.[12] Trauma and cold induces the degeneration of collagen with thinning of epidemis in genetically predisposed individuals. Our patients did not have any systemic disease, indicating that systemic disease plays no role in the etiology of familial variety of RPC. Histopathologically, focal disruptions of the epidermis expelling collagen bundles and degenerated inflammatory cells occur in RPC.[13,14] Our patients showed features that are consistent with RPC on histopathological examination and special staining for collagen.

Lesions are usually self healing without any treatment but often recur. Various treatments, including isotretinoin, allopurinol, methotrexate, doxycycline, phototerapy, emollients and oral antihistamines, were tried.[3] Our patients showed good response to oral isotretinoin and topical tretinoin combined with emollients, but long-term treatment is required. Retinoids may have a stabilizing effect on keratinocytes, thereby preventing the focal damage of collagen and necrolysis of epidermis.
